RETRACTED

# Quetiapine Combined with Sodium Valproate in Patients with Alzheimer's Disease with Mental and Behavioral Symptoms Efficacy Observation

**DOI:** 10.1155/2022/1278092

**Published:** 2022-01-17

**Authors:** Zhihua Zhang, Jiating Xu, Penghao Xu, Wenjun Liu, Xianyan He, Kedeng Fu

**Affiliations:** Senile Psychiatry Department, The Third Hospital of Quzhou, Quzhou 324000, Zhejiang, China

## Abstract

Quetiapine combined with sodium valproate is an effective and more suitable drug treatment for Alzheimer's disease. At present, there are relatively few studies on the combined action mechanism of these two drugs. This study has certain practical value. Alzheimer's disease is a multifaceted, highly genetically heterogeneous neurodegenerative disease. The main clinical manifestations are memory loss, abnormal mental behavior, and loss of various cognitive functions. In order to improve the symptoms of patients with Alzheimer's disease, especially those with mental symptoms, this article combines quetiapine and sodium valproate, two commonly used drugs for the treatment of mental illnesses, and applies them to different levels of Alzheimer's and observes the results of the combination's curative effect. This article introduces Alzheimer's disease and its potential mental behaviors in the method section, and it also introduces the mechanism of action of quetiapine and sodium valproate. For the algorithm, this paper introduces a data mining algorithm to understand the effect of drug efficacy. In the experimental part, firstly, it introduces the experimental objects, the proportion of medicines, and the statistical methods. Secondly, this article covers adverse reactions, inflammatory factors and vascular endothelial indicators, Alzheimer's disease performance, MOAS score, treatment effect evaluation, and satisfaction surveys. It can be seen from the experiment that, in mental behavior, the experimental group decreased from 8.2 before treatment to 0.5, and the control group decreased from 7.1 before treatment to 2.6. It can be seen that the scores of the experimental group changed after receiving the treatment of quetiapine combined with sodium valproate.

## 1. Introduction

Dementia refers to acquired and persistent cognitive impairment syndromes caused by brain dysfunction. Knowledge refers to the process by which the human brain transforms into internal mental activities through processing, receives external information, and acquires knowledge, including memory, language, performance, visual space, calculation, and cognitive judgment. With the rapid increase in the elderly population, the number of patients with dementia has increased significantly, and Alzheimer's disease is the most common dementia. Quetiapine is used for various types of schizophrenia. Not only is it effective for positive symptoms of schizophrenia, but also it has a certain effect on negative symptoms; it can also alleviate emotional symptoms related to schizophrenia such as depression and anxiety and cognitive deficit symptoms. Sodium valproate is a broad-spectrum antiepileptic drug. It is an inhibitor of GABA transaminase in the brain, which can slow down the catabolism of GABA; at the same time, it can increase the activity of glutamate decarboxylase and increase the production of GABA, thereby increasing the GABA content of inhibitory synapses in the brain, and can increase postsynaptic inhibition. The membrane is responsive to GABA, thereby enhancing GABAergic postsynaptic inhibition. It does not inhibit the discharge of epileptic lesions, but it can prevent the spread of abnormal discharges of the lesions.

RETRACTED

The International Society of Geriatric Psychiatry defines the psychological and behavioral symptoms associated with Alzheimer's disease as a group of common abnormal and pathological symptoms in dementia patients. Patients with dementia show different forms of psychological and behavioral symptoms, some show indifference, and some show enthusiastic behavior. Psychological behavioral symptoms are an important part of the clinical manifestations of dementia, covering almost all types of psychological symptoms. Not all mental behaviors occur at the same time, and they often occur individually or as a combination of multiple symptoms. In addition, patients with Alzheimer's disease may have mental disorders such as behavioral disorders, aggression, anxiety, and delusions, but their intelligence gradually declines, which further aggravates the damage to their social functions and increases the economic and spiritual burden of the family.

At present, there are many methods for Alzheimer's disease, but they are still not satisfactory, and there is no drug for pathological Alzheimer's disease. At the same time, the options for behavioral symptoms are very limited, and it is still a difficult treatment in the world. Although many antipsychotic drugs such as risperidone and olanzapine can significantly improve the mental and behavioral symptoms of Alzheimer's disease, they are well tolerated. But there are some research strategies for drugs in the treatment of mental behavior. There is no significant difference from depression, and it is easy to increase the risk of death of patients. It is necessary to always pay attention to the mental symptoms, cognitive function, and safety status of patients with Alzheimer's disease, observe the improvement effects and adverse reactions of their condition, and provide reference for the clinical treatment of Alzheimer's disease.

RETRACTED

Many scholars have done related research on the topic of quetiapine combined with sodium valproate in the treatment of Alzheimer's disease. Sperling RA further clarified the relationship between the pathological cascade of Alzheimer's disease and the appearance of clinical symptoms. The scholar conducted research on Alzheimer's disease but did not propose an improvement method [1]. Phillips et al. investigated that emotion perception problems were independent of cognitive function and the variance of emotion prediction to predict quality of life. The scholar conducted a group study on the affective disorder of patients with Alzheimer's disease from the perspective of quality of life, but related indicators were lacking [2, 3]. Fleisher et al. hoped to develop biomarkers of the disease and even identify abnormal brain structures or functions before cognitive decline. The scholar performed data processing on Alzheimer's therapeutic drugs but did not compare other drugs [4]. Stephenson et al. compared quetiapine with patients treated with typical antipsychotics and clozapine previously studied. Quetiapine treatment leads to marginal selective *D* (2)/*D* (3) blockade similar to clozapine and significantly higher than typical antipsychotics. The experimental data indicate that edge-selective *D* (2)/*D* (3) receptor blockade is important for atypical drug effects. The authors conducted research on quetiapine but did not incorporate some mechanism of action [5]. The purpose of Abolghasem et al.'s study was to determine the frequency of changes in biochemical and bone mineral density in adults receiving valproic acid and carbamazepine. In a cross-sectional study, adults (20–50 years of age) with epilepsy who had received valproic acid or carbamazepine for at least 2 years were evaluated. In addition, after starting CBZ and VPA treatment, all patients with epilepsy can consider calcium supplementation. The scholar applied sodium valproate to patients with epilepsy but did not propose a prospect of application [6, 7]. In order to evaluate the achievement of medical treatment and treatment target parameters of patients with ischemic heart disease (IHD) during the 3–5-year follow-up period after coronary artery bypass surgery, Barbarash OL obtained the initial sample (*n* = 680) from the registration of coronary artery bypass surgery. 111 men were selected for this study. Clinical practice data show that the quality of basic and antiangina treatment for IHD patients after CABG is insufficient. The scholar designed experiments to study drug treatment but did not propose an improved plan [8]. In Andrzej et al.'s study, patients received 20 years of prospective observation after completing SIT to determine its effectiveness. The scholars conducted research on treatment observation but did not propose a related algorithm [9].

RETRACTED

Based on the two drugs of quetiapine and sodium valproate, this article observes and studies the therapeutic effects of patients with Alzheimer's disease with psychobehavioral symptoms. This article introduces Alzheimer's disease and its possible mental behaviors in the method section, and it also introduces the mechanism of action of quetiapine and sodium valproate. On the algorithm, this paper introduces a data mining algorithm to understand the effect of drug efficacy. In the experimental part, this article analyzes the various aspects of research from adverse reactions, inflammatory factors and vascular endothelial indicators, Alzheimer's disease performance, MOAS score, treatment effect evaluation, and satisfaction survey. The innovation of this article is that it combines quetiapine and sodium valproate, two drugs for the treatment of mental illness, and analyzes a variety of scoring indicators related to Alzheimer's disease. The level of daily life is analyzed [10, 11]. Using the logistic regression function in the data mining algorithm to linearly process the data, the two drugs, quetiapine and sodium valproate, were used to score the therapeutic effects of MOAS, PANSS, and BPRS during the treatment experiment. Compared with traditional drug therapy, the drug therapy of quetiapine combined with sodium malate proposed in this article is superior to traditional drug therapy in terms of safety and adverse reactions and can effectively reduce the adverse risks of drug therapy.

## 2. Curative Effect of Quetiapine Combined with Sodium Valproate on Patients with Alzheimer's Disease Accompanied by Mental and Behavioral Symptoms Observation Method

### 2.1. Alzheimer's Disease

Alzheimer's disease (AD) is one of the most common neurodegenerative diseases that cause dementia. Its clinical manifestations are progressive memory loss, accompanied by cognitive decline. The term Alzheimer's disease comes from pathologist Alois Alzheimer. In 1906, a brain examination of a patient found that there were a large number of senile plaques in his brain, and the disease caused by this characteristic senile plaque was officially named AD (8-9). Alzheimer's disease is the most important and common type of disease. It is mainly caused by widespread senile plaques in the cerebral cortex and tangles of fibrous filaments in the brain tissue, resulting in the degeneration of brain function. Its pathological features mainly include senile plaques formed by amyloid aggregation, neurofibrillary tangles (NFTs) formed by hyperphosphorylation of Tau protein, and neuron loss and synaptic dysfunction. This kind of disease mainly occurs in the elderly, especially in the elderly above 65 years of age. According to the age of onset of patients, it can be divided into Alzheimer's disease, of which the senile dementia patients account for the majority [12]. Under the electron microscope, the patient's NFT is composed of a straight nerve wire and a double-stranded spiral nerve wire. Many studies have shown that NFT is related to abnormal cytoskeleton composition. Immunohistochemical staining confirmed the presence of phosphorylated and nonphosphorylated neurofilaments and microtubule-associated protein II (MAPII). Alzheimer's disease is a persistent type of disease. which is mainly caused by underlying neuropathy and neurochemical changes in the brain and causes the gradual deterioration of cognitive function, decline in memory, learning ability, concentration, and judgment, problems with time and space, communication difficulties, decreased personal hygiene and self-care ability, inappropriate social behaviors, and personality changes. Recent memory loss is one of the most common early symptoms of Alzheimer's disease; the most common and prominent early symptoms are decreased calculation ability, decreased understanding and expression ability, decreased time concept, decreased ability to recognize ways, and large emotional changes.

RETRACTED

At present, it is clear that the brain of AD has the following main pathological features: (1) high-density senile plaques appear outside the cells; (2) a large number of neurofibrillary tangles appear in neurons; (3) the neuritis reaction that occurs in the brain. Among them, the main component of senile plaques is amyloid *β* protein (A*β*), which is produced by *β*-amyloid precursor protein (APP) by *β*-secretase and *γ*-secretase. A*β* is a peptide with strong resistance to protein degradation, consisting of 37 to 43 amino acids, and its isomers A*β*1-40 and A*β*1-42 are the most common. A*β*1-42 is currently considered the most toxic. Due to the physical and chemical properties of A*β*1-42, the configuration is *β*-sheets, which are easy to aggregate and form the core of amyloid plaques. At the same time, A*β* is also a component of amyloid neuroinflammatory plaques. Studies have shown that the number of NFTs is positively correlated with the severity of dementia [13, 14]. It is worth noting that there is an interaction between A*β* in the brain and highly phosphorylated tau protein. The result is to further accelerate the damage of neurons and further activate glial cells in the form of self-reproduction, resulting in a neuroinflammatory response and eventually forming a vicious circle of disease. In short, the accumulation of A*β* in the brain, abnormal accumulation of highly phosphorylated tau protein, and neuroinflammation constitute the main pathological features of AD and pose a great threat to the survival of neurons and their functional activities. Amyloid deposition was once considered to be the main pathological factor of AD, which mainly involved the senile plaques formed by A*β*1-42 and A*β*1-40 deposited outside the cell. Studies have shown that amyloid precursor protein (APP) is closely related to AD disease. Mature A*β*1-42 and A*β*1-40 continue to accumulate outside the cell and cannot be removed, eventually forming senile plaques, affecting normal brain functions. In addition, studies have found that there are varying degrees of amyloid aggregation in the brains of AD patients [15, 16].  Figure 1 shows how Alzheimer's disease works.

RETRACTED

Alzheimer's disease, a degenerative disease of the nervous system, is usually caused by a variety of factors. In the early stage, there are mainly episodic memory impairment and memory loss of recent events. As the disease progresses, it will gradually develop. Memory loss, work, and learning new knowledge will gradually increase [17]. And there will be cognitive impairments in many other areas such as decreased social contact. The typical symptoms of histopathology are amyloid plaques and neurofibrillary tangles. Studies have shown that different areas of the brain of patients with Alzheimer's disease, especially the temporal lobe and corpus callosum, are damaged to varying degrees, which further impairs the memory and learning ability of patients with Alzheimer's disease. The psychological and behavioral symptoms of Alzheimer's disease include the following: agitation/aggression, abnormal motor behavior, and sleep disturbance. Stimulus is the inappropriate behavior of tongue, voice, and movement and cannot be explained by the patient's specific needs or ecstasy. The frequency of AD stimulation is higher than that of MCI. The behavioral symptoms of upset patients are usually more severe. All behavioral symptoms of AD patients are more severe than those of AD patients without stimulation, but the circadian rhythm disorders of MCI patients are more severe than those of AD patients. Nonaggressive behavior language is the most common, and physical aggressive behavior is the most difficult for nursing staff to deal with [18, 19]. The higher the incidence of BPSD (especially agitation/aggressive behavior) is, the higher the degree of general dementia is.  Figure 2 shows the brain changes in Alzheimer's disease.

RETRACTED

### 2.2. Quetiapine

Quetiapine is an atypical antipsychotic, which mainly blocks dopamine D2 and serotonin receptor type 2 (5-HT2), acting on dopamine D1, D4, histamine receptor type 1 (H1), and adrenergic receptor. Many studies have shown that quetiapine has a positive effect on the positive and negative symptoms of schizophrenia, which can improve the cognitive function of patients, thereby improving the social adaptability and individual psychology of patients, which can be seen to promote physical and mental recovery [20, 21]. First of all, children and adolescents do not have precise regulations on the dosage of this drug, and this drug has not been formally approved. The side effects caused by it are too large, and the physique of children and adolescents is relatively weak.

Quetiapine fumarate is the most commonly used type of MA. It has a good effect on both positive and negative symptoms of schizophrenia. It can bind to multiple receptors in the brain. The drug has a significantly higher affinity for serotonin receptors than dopamine receptors and has a specific binding effect on the dopamine system of the limbic lobe and midbrain cortex, making its side effects on cranial nerves and endocrine significantly less than classic antipsychotic drugs (haloperidol, chlorpromazine, etc.); it has a small effect on the dopamine receptors of the substantia nigra striatum, so extrapyramidal side reactions rarely occur; it has a weak effect on the dopamine system in the nodular funnel, thus avoiding the occurrence of hyperprolactinemia. Based on the above advantages, patients have good compliance and high satisfaction when using quetiapine fumarate treatment, which increases the therapeutic effect and greatly improves the quality of life of patients [22, 23]. Therefore, the drug is widely used to treat patients with long-term schizophrenia, especially those elderly patients who have more side effects when using other drugs.

### 2.3. Sodium Valproate

Sodium valproate (VPA) is a histone deacetylase inhibitor, mainly used in medicine to treat epilepsy and bipolar disorder. The current research on histone deacetylase inhibitors is mainly focused on the level of regulation of histone modification. Typical forms of histone modifications include methylation, acetylation, phosphorylation, and extensive. Acetylation is a very common and important histone modification used to regulate gene expression and chromatin structure [24, 25]. Martin In eukaryotes, the homeostasis of acetylation is essential for maintaining normal cell functions. The process is based on the participation of two enzymes, histone acetyltransferase and histone deacetylase.

RETRACTED

Currently, the bioavailability of oral VPA exceeds 80%. Current experiments show that VPA can affect the aminobutyric acid system, inhibit ketoglutarate dehydrogenase, *γ*-aminobutyric acid transaminase, and semialdehyde oxidase dehydrogenase, and increase *γ*-*α* acid. This suggests that VPA may affect brain metabolism by activating GABA receptors and blocking sodium ion channels, thereby regulating the treatment of calcium and potassium ions and the delivery of dopamine and serotonin. Applicable conditions of sodium valproate are as follows: (1) use with caution in patients with acute and chronic hepatitis; (2) use with caution in patients with allergies; (3) disable for patients with severe hepatitis or family history; (4) and disable for patients with urea cycle disorders.

### 2.4. Data Mining Model for Drug Therapy

The main metabolites in human plasma do not have obvious pharmacological activity. Eating has no significant effect on the bioavailability of quetiapine. Since sodium valproate inhibits r-aminobutyric acid transaminase, the concentration of inhibitory neurotransmitter r-aminobutyric acid in the brain is increased to achieve the antiepileptic purpose. By combining the two drugs of quetiapine and sodium valproate and mining and integrating the big data of their therapeutic effects, it is helpful to understand the effect of the combination. In this regard, this article introduces some nonintegrated learning prediction models.

#### 2.4.1. Support Vector Machine

Support vector machine is a two-classification model, and its basic model is defined as the linear classifier with the longest distance in the feature space. The learning strategy is to maximize the space between the classes to obtain a plane. First define some data points and set their category to *n*. From this, a kind of hyperplane can be found in the data space, which is expressed as follows:

(1) $$\begin{array}{c} g\left(m\right)=\mathrm{sgn}\left\{hm+c\right\}. \end{array}$$

The greater the distance between the data point and the hyperplane is, the more reliable the classification is, and vice versa. The function interval between the data point (*m*, *n*) and the hyperplane is

(2) $$\begin{array}{c} \frac{Ν}{\chi }=n\cdot \left(h\cdot m+c\right). \end{array}$$

In addition, some constraints need to be added to the normal vector *h* of the hyperplane, for example, *h* = 1, so that the interval is determined. The interval after the constraint is added is the relationship between the geometric interval function interval and the geometric interval as follows:

(3) $$\begin{array}{c} \chi =\frac{Ν/\chi }{\left\|h\right\|}. \end{array}$$

Solve the following constrained optimization problem:

(4) $$\begin{array}{c} \underset{h,c}{\max}=\chi ,\\ s.t.\;n_{x}\left(\frac{h}{\left\|h\right\|}\cdot m_{x}+\frac{c}{\left\|h\right\|}\right)\geq \chi ,x=1,2,\ldots ,M. \end{array}$$

Taking into account the geometric interval and function interval, the above formula is modified as

(5) $$\begin{array}{c} \underset{h,c}{\max}=\frac{\hat{\chi }}{\left\|h\right\|},\\ s.t.\;n_{x}\left(h\cdot m_{x}+c\right)\geq \hat{\chi },x=1,2,\ldots ,M. \end{array}$$

Since the value of the function interval does not affect the result, we can consider the optimization problem supported by the linear separable vector learning machine.

(6) $$\begin{array}{c} \underset{h,c}{\min}=\frac{1}{2}{\left\|h\right\|}^{2},\\ s.t.\;n_{x}\left(h\cdot m_{x}+c\right)-1\geq \hat{\chi },x=1,2,\ldots ,M. \end{array}$$

Define the kernel function, and use the kernel function to map the data in the high-dimensional space, so that the indivisible data in the original space can be divided in the high-dimensional space:

(7) $$\begin{array}{c} g\left(m\right)=\mathrm{sgn}\left\{\overset{r}{\underset{x=1}{\sum }}\varepsilon_{x}n_{x}L\left(m_{x},m\right)+c\right\}. \end{array}$$

RETRACTED

#### 2.4.2. K-Nearest Neighbors

K-nearest neighbor (KNN) method is one of the commonly used classification methods. The input is the features of the training set, the output is the classification result, and the classification result can be multiclass. First, *m* is assumed to be a new data point. The *K* point found in the data set *G* that is the nearest neighbor to *m* is the domain *Y*_*K*_(*m*), and the majority vote on it is

(8) $$\begin{array}{c} n=\arg\underset{b_{y}}{\max}\sum_{m_{y}\in J_{K}\left(m\right)}X\left(m_{x}=b_{x}\right),x=1,2,\ldots ,M;y=1,2,\ldots ,N. \end{array}$$

We have that *P* is the indicator function. When *m*_*x*_=*b*_*x*_, we have *P* = 1.

#### 2.4.3. Logistic Regression

Before mentioning logistic regression, it is necessary to mention linear regression. Linear regression is a statistical analysis method used to determine the correlation between variables. Strictly speaking, there is a difference between the statistical field and the machine learning field, but linear regression is a popular method that both fields prefer.

First establish a hypothetical function model:
  (9) $$\begin{array}{c} l_{\sigma }\left(m\right)=\sigma_{0}m_{0}+\sigma_{1}m_{1}+\sigma_{2}m_{2}+\sigma_{3}m_{3}+\ldots +\sigma_{j}m_{j}. \end{array}$$
Second, establish the loss function as
  (10) $$\begin{array}{c} Y\left(\sigma \right)=\frac{1}{2}{\overset{i}{\underset{x=1}{\sum }}\left(l_{\sigma }\left(m_{x}\right)-n_{x}\right)}^{2}. \end{array}$$
Third, use stochastic gradient descent to find the parameters:
  (11) $$\begin{array}{c} \frac{\partial Y\left(\sigma \right)}{\partial \sigma_{y}}=\overset{i}{\underset{x=1}{\sum }}m_{x}\left(l_{\sigma }\left(m_{x}\right)-n_{x}\right),\\ \sigma_{y}=\sigma_{y}-\lambda \frac{\partial Y\left(\sigma \right)}{\partial \sigma_{y}}. \end{array}$$

In the above equation, *λ* is the learning efficiency, which needs to be kept in an appropriate interval. Let *M* be a continuous random variable and obeying the logistic distribution means that *M* has the following distribution function and density function:

(12) $$\begin{array}{c} G\left(m\right)=Q\left(M\leq m\right)=\frac{1}{1+e^{-\left(m-v\right)/\vartheta }},\\ g\left(m\right)=G^{\prime }\left(m\right)=\frac{e^{-\left(m-v\right)/n}}{n\cdot \left(1+e^{-\left(m-v\right)/\vartheta }\right)}. \end{array}$$

In the above equation, *v* is the position parameter and *ϑ* is the shape parameter.

RETRACTED

Logistic regression model generally refers to a binary logistic regression model, which is a classification model. The original model is a binary classification model, and even a disproportionate data set can be transformed into a polynomial regression logistic model (similar to SVM). This model can be expressed as

(13) $$\begin{array}{c} Q\left(N=1|m\right)=\frac{\exp\left(h\cdot m+c\right)}{1+\exp\left(h\cdot m+c\right)},\\ Q\left(N=0|m\right)=\frac{\exp\left(h\cdot m+c\right)}{1+\exp\left(h\cdot m+c\right)}. \end{array}$$

For the logistic regression model, modeling is still carried out in the above-mentioned way. First establish a hypothetical function:

(14) $$\begin{array}{c} Q\left(N=1|m\right)=\frac{1}{1+e^{-h_{\sigma }\left(m\right)}}=f\left(l_{\sigma }\left(m\right)\right). \end{array}$$

The loss function of the regression can be determined by estimating the maximum probability and estimating the model parameters.

(15) $$\begin{array}{c} Q\left(N=1|m\right)=\pi \left(m\right),Q\left(N=0|m\right)=1-\pi \left(m\right). \end{array}$$

The likelihood function is

(16) $$\begin{array}{c} \prod_{x=1}^{J}\left[\pi {\left(m_{x}\right)}^{n_{x}}\right]{\left[1-\pi \left(m_{x}\right)\right]}^{1-n_{x}}. \end{array}$$

The log-likelihood function is

(17) $$\begin{array}{c} D\left(h\right)=\sum_{x=1}^{J}\left[n_{x}\log\;\pi \left(m_{x}\right)+\left(1-n_{x}\right)\log\left(1-\pi \left(m_{x}\right)\right)\right]. \end{array}$$

In addition, genetic algorithm has the implicit parallelism, which is easy to combine with other models and other properties, so that it can be used in data mining. Decision tree is an algorithm commonly used in predictive models. It can find some valuable and potential information by classifying a large amount of data purposefully. These methods have advantages in data processing.

RETRACTED

## 3. Quetiapine Combined with Sodium Valproate on Patients with Alzheimer's Disease Accompanied by Mental and Behavioral Symptoms Efficacy Observation: Experiment and Results

### 3.1. Experiment Object

The experimental subjects in this article are all elderly patients who were hospitalized in a hospital from 2019 to 2020. A total of 100 cases, 64 males and 36 females, were randomly divided into experimental and control groups, with 50 people in each group and no other significant ones.

### 3.2. Drug Ratio

The dosage of sodium valproate sustained-release tablets (Derbakin: 500 mg/tablet = 30 tablets/bottle) is as follows: the initial oral dose is 250 mg, according to the patient's clinical manifestations and drug tolerance, gradually increase the dose to 1.0∼1.25 g/d within 1 week, and continue treatment for 15 weeks. Preparation of quetiapine standard solution is as follows: Weigh 11.56 mg of the nearest quetiapine fumarate (quetiapine 10.04 mg), dissolve it in methanol, and place it in a 10 ml volumetric flask to obtain a quetiapine concentration of 1.004 mg/mL the standard stock solution. The stock solution was diluted with methanol to obtain a series of working solutions containing quetiapine at 10.04, 20.08, 100.4, 502.0, 1004, 2008, and 5020 ng/mL.

### 3.3. Statistical Methods

After all the data are completed, they are sorted in Excel. The measurement data was analyzed and compared with *t*-test. The count data were analyzed through a secondary study and Spearman correlation analysis to analyze the correlation between the dose of quetiapine and side effects.

### 3.4. General Information

Table 1 shows the general conditions of the patients. It can be seen that the age distributions of mild, moderate, and severe patients are relatively similar, and Alzheimer's disease is generally distributed around 70 years of age.

### 3.5. Adverse Reactions

Common symptoms of adverse reactions include hypotension, abnormal body function, rapid heartbeat, constipation, dry mouth, and lethargy. From Figure 3, we can see that, in the experimental group, lethargy and abnormal liver function accounted for the largest proportion, while in the control group, lethargy, hypotension, and heart rate acceleration accounted for the largest proportion. This can be seen through the realization of quetiapine combined with sodium valproate drug treatment, which reduces the occurrence of some adverse reactions.

Figure 4 shows the comparison of NPI between the two groups of patients. NPI refers to some of the above-mentioned adverse reactions. Here, the time after treatment is subdivided into the first, second, third, fifth, tenth, twelfth, fifteenth, and twenty-fifth weeks. The research and analysis of treatment results are carried out in the 25th week after treatment.

RETRACTED

### 3.6. Manifestations of Alzheimer's Disease

BEHAVE is Alzheimer's behavioral pathology table, which includes patient behaviors such as paranoia, hallucinations, aggression, affective disorders, behavioral disorders, and anxiety. After receiving relevant treatment, the score will be reduced as shown in Figure 5.

### 3.7. Inflammatory Factors and Vascular Endothelial Indicators

As shown in Figure 6, there was no significant difference in inflammatory factor levels and vascular endothelial index. The levels of IL-1 and TNF were lower than those before treatment.

### 3.8. MOAS Score Comparison

It can be seen from Table 2 that the MOAS score is an assessment of the risk of violence for patients with mental illness.

### 3.9. Evaluation of Treatment Effect

Figure 7 shows the comparison of the effects after 2 weeks and 4 weeks of treatment.

Figure 8 shows the PANSS of the experimental group, that is, the comparison of the positive and negative symptom scale scores. This score will decrease with the increase of treatment time. It can be seen from Figure 7 that, during the six weeks of treatment, the positive symptoms and psychopathology have been maintained at a relatively high level. As the treatment time increases, the positive symptoms, negative symptoms, and psychopathology are all significantly reduced.

Table 3 shows the BPRS score reduction rate before and after treatment. The difference was statistically significant after the first, second, and third weeks of treatment. In the first week, the experimental group had a greater degree of reduction of 0.14, while the control group had a reduction of 0.032. In the experimental group, there was no statistical significance in the fifth and tenth weeks of treatment.

### 3.10. Satisfaction Survey

As shown in Figure 9, the family members of the experimental group and the control group were satisfied with the combination medication. It can be seen from the figure that 59.63% of the family members in the experimental group are satisfied with the combination medication, and 39.74% are satisfied with the combination medication. The family members of the control group were satisfied with the treatment.

## 4. Discussion

The incidence of mental behaviors associated with Alzheimer's patients remains high, and it occurs and develops throughout the course of the disease and will further develop as the disease worsens. The biggest problem in the treatment and management of mental behavior is early recognition. The early symptoms of dementia are not easy to detect, which delays treatment. However, once Alzheimer's patients show symptoms of mental behavior, it means that Alzheimer's development is more serious. Psychiatrists must conduct systematic, comprehensive, and professional diagnosis and evaluation as soon as possible, make professional judgments on Alzheimer's disease, classify mental behavior, and optimize diagnosis and treatment plans based on the gender of the disease, the type of dementia, and the type of mental behavior. In the drug treatment of Alzheimer's associated mental behavior, the treatment of Alzheimer's should be considered first. Alzheimer's is the foundation of the existence and development of mental behavior. Only when Alzheimer's is treated systematically can it be treated. Fundamentally cure mental behavior; the preferred optimal management method for mental behavior is nonpharmacological intervention therapy, such as rehabilitation therapy and music therapy, strengthening cognitive training and functional recovery. The use of antipsychotics should be cautious. It must be used with caution when nonpharmacological interventions are ineffective. Of course, in the face of moderate-to-severe mental behaviors, appropriate antipsychotics can be used for symptomatic treatment in order to control symptoms. First of all, the patient can be inspected on time for a long time, and the pathology can be judged according to the guidelines. As the patient's condition improves, the dose can be gradually reduced while improving his physical fitness in another way. Improve function; before using drugs, it should be kept in mind that as the body degenerates and organs age, not only are psychiatric patients old and weak, but also they have many underlying diseases, such as coronary heart disease, diabetes, high blood pressure, hyperlipidemia, and other diseases. It is common, and dementia patients have poor cardiopulmonary function, decreased liver and kidney metabolism, and even liver disease. Therefore, after the drug enters the human body, it is easy to accumulate, which leads to an increase in blood drug concentration and the risk of sudden death in severe cases. Moreover, antipsychotic drugs may not only damage cognitive function and induce epilepsy or Parkinson's disease but also even cause death.

RETRACTED

Sodium valproate increases the content of aminobutyric acid in the brain by inhibiting aminobutyric acid transaminase and semialdehyde electrode hydrogenase in the brain, thereby reducing the stimulation of neurons. This is a common mood stabilizer in clinical practice. Low-dose sodium valproate has a therapeutic effect on the psychological and behavioral symptoms of dementia, with few side effects. Due to the weakened metabolic capacity of the elderly, the use of a smaller dose of quetiapine can effectively control the symptoms of Alzheimer's and obtain a satisfactory drug treatment effect. Studies have found that the combination of quetiapine and sodium valproate sustained-release tablets for the treatment of patients with Alzheimer's disease is significantly better than sodium valproate sustained-release tablets. This result can be used as a reference for future clinical drug treatment. The study also found that the BEHAVE, PANSS, MOSA, and BPRS scores of the experimental group were better than those of the control group. Quetiapine is used in combination with sodium valproate to treat Alzheimer's disease with psychological and behavioral symptoms.

## 5. Conclusion

The psychological and behavioral symptoms of Alzheimer's disease patients worsen the condition, which further threatens the personal safety of the patients and the people around them and increases the burden on the family and society. At all stages of the disease, psychological and behavioral symptoms such as agitation/aggression, hallucinations, sleep disturbances, irritability, and anxiety will appear. First of all, the drug can alleviate symptoms such as anxiety and depression related to schizophrenia. Since this drug is mainly aimed at the positive mental symptoms of schizophrenia, it has a certain inhibitory effect. After taking the drug, patients will experience symptoms such as easy sedation, drowsiness, and weakness in limbs. In severe cases, it may have hypotension. This study is to conduct experiments on elderly people who actually suffer from Alzheimer's disease combined with scientifically based drugs. The data is reliable and the experiment is risk-free. This article aims to observe the efficacy of quetiapine combined with sodium valproate in the treatment of Alzheimer's disease with mental behavior. This article analyzes from different research perspectives such as adverse reactions, inflammatory factors and vascular endothelial indicators, Alzheimer's disease manifestations, MOAS scores, evaluation of treatment effects, and satisfaction surveys. It is concluded that, in terms of mental behavior, the experimental group decreased from 8.2 before treatment to 0.5, and the control group decreased from 7.1 before treatment to 2.6. It resulted in a better effect of the drug treatment method compared to the traditional method. The treatment effect is significant in improving mental behavior symptoms, can effectively improve cognitive status, and has no obvious adverse reactions. It is expected to become the main drug for the treatment of Alzheimer's disease and provide scientific theoretical basis for clinical application of the prevention and treatment of Alzheimer's disease, to further explore modern treatment methods for Alzheimer's disease. The shortcoming of this article is that it has not studied whether the simultaneous use of quetiapine and sodium valproate has any effect on psychosis and behavioral symptoms other than Alzheimer's disease, as well as the effect of different doses of quetiapine and sodium valproate on mental behavior. No relevant research has been done on the degree. It is hoped that, with the research on mental illness and related therapeutic drugs, the research conclusions of this article can be further optimized.

RETRACTED

## Figures and Tables

**Figure 1:** How tau works on Alzheimer's.

**Figure 2:** Changes in the brain during dementia.

**Figure 3:** Comparison of adverse reactions between the two groups.

**Figure 4:** Changes and comparison of NPI total scores between the two groups of patients at different time points.

**Figure 5:** BEHAVE score before and after treatment in the two groups. (a) Test group. (b) Control group.

**Figure 6:** Comparison of inflammatory factors and vascular endothelial index levels before and after treatment. (a) Test group. (b) Control group.

**Figure 7:** Comparison of treatment effects after 2nd and 4th weeks. (a) Two weeks later. (b) Four weeks later.

**Figure 8:** PANSS score comparison.

**Figure 9:** Comparison of family satisfaction.

**Table 1:** List of patients.

	Mild Alzheimer's disease	Moderate Alzheimer's disease	Severe Alzheimer's disease
Age	73.234	72.145	70.463
Gender	32 (52.1)	22 (38.3)	10 (37.8)
Years of education	11.43	7.43	5.47
Course of disease	29.45	31.66	57.89
Family history	17	12	6

**Table 2:** Comparison of MOAS scores between the two groups before and after treatment.

Group	Before treatment	1 week of treatment	3 weeks of treatment	5 weeks of treatment
Test group	14.23	8.52	6.34	4.52
Control group	13.87	11.12	8.32	6.15
*t*	0.51	3.12	3.05	2.32
*P*	>0.05	<0.01	<0.01	<0.05

**Table 3:** Comparison of BPRS score reduction between the two groups.

Group	Before	1-week reduction rate	2 weeks' reduction rate	3 weeks' reduction rate	5 weeks' reduction rate	10 weeks' reduction rate
Test group	44.87	0.14	0.18	0.29	0.36	0.48
Control group	44.94	0.032	0.103	0.13	0.25	0.34
*t*	0.4546	9.214	5.187	8.682	1.102	0.4982
*P*	0.6134	<0.0001	<0.0001	<0.0001	0.2115	0.6144

## Data Availability

The data that support the findings of this study are available from the corresponding author upon reasonable request.
